# Sleep Status and Menstrual Problems among Chinese Young Females

**DOI:** 10.1155/2021/1549712

**Published:** 2021-10-25

**Authors:** Hong He, Xiaoxuan Yu, Tingjia Chen, Fei Yang, Min Zhang, Hui Ge

**Affiliations:** ^1^Health Care and Physical Examination Center, The First Affiliated Hospital, Sun Yat-sen University, Guangzhou 510080, China; ^2^Department of Epidemiology, School of Medicine, Jinan University, Guangzhou 510630, China

## Abstract

**Background:**

The association between sleep disturbance and the menstruation in the young women population has been scarcely studied. The aim of this study is to assess the association between sleep status and phase of the menstrual cycle in healthy, young, ovulating women.

**Methods:**

This cross-sectional study used the data collected from healthy young, ovulating Chinese females from September to December 2018. The association was analyzed by using linear regression and binary logistic analyses.

**Results:**

2260 women aged 17 to 30 were included in the analysis. The average sleep duration of the respondents was 7.24 hours (SD = 0.92). 61.7% of them admitted that they were accompanied by at least one of sleep symptoms including difficulty initiating sleep, difficulty maintaining sleep, dreaminess, early morning awakening, and somnolence. Sleep quality was significantly associated with dysmenorrhea (OR [95%CI] = 1.74 [1.40-2.17], *P* < 0.001) and self-awareness menstrual regularity (OR [95%CI] = 1.29 [1.06-1.56], *P* = 0.011).

**Conclusion:**

This study found that poor sleep quality is significantly associated with dysmenorrhea and self-awareness menstrual irregularity among healthy, young, ovulating, Chinese females.

## 1. Background

Many women experience mense-related health problems during their reproductively fertile years, such as menstrual cycle irregularity, menstrual pain, heavy menstrual bleeding, and premenstrual syndrome [1]. For instance, about 25% of women in the world suffer from menstrual pain, which leads to work productivity loss [2].

Menstrual symptoms and menstrual cycle irregularity can be caused by diseases, such as breast cancer, type 2 diabetes, cardiovascular disease, osteoporosis, and infertility [3–6]. Besides, various physical and mental conditions and health-related lifestyles could also affect menstrual health [7].

Recently, sleep disturbance has been associated with menstrual disorder in adults. As well known, good quality sleep is essential for our optimal daytime performance of various daily tasks, whereas inadequate sleep causes daytime malfunctioning, psychological and behavioral problems, and physical disorder [8]. 10-35% of the general population are affected by insufficient or nonrestorative sleep, among which women have higher prevalence of sleep disturbance than men [9–11].

Several studies imply that sleep may correlate with reproductive function in females [12]. Baker and Driver infer that circadian disruption such as sleep-wake disorders may disturb the menstrual cycle [13]. A population-based cross-sectional study conducted in Korea found that female adolescents with menstrual cycle irregularity have significantly shorter sleep duration and higher depressive mood than those without menstrual cycle irregularity [14].

However, the association between the sleep disturbance and the menstruation of females in China has not been studied yet. Therefore, this work was aimed at investigating the relationship of the sleep pattern and the menstruation to healthy, young, ovulating women in China.

## 2. Methods

### 2.1. Data Collection

The cross-sectional study achieved the data by e-questionnaire among nationwide females. In October-November, 2018, a total of 2517 e-questionnaires were returned. The questionnaire was completed to assess female basic information, sleep conditions, and menstrual conditions. Before filling out the questionnaire, participants were instructed to inform that this research was anonymous and their engagement was voluntary without any rewards or penalties. The study was approved by the research ethics committee of Jinan University.

### 2.2. Study Covariates

Basic information and lifestyle features of subjects were asked. Those were selected for this study as covariates included female's age, body mass index (BMI), physical activity, monthly expenditure, and medication history. These confounding factors had the associations of these variables with sleep and menstruation in previous research [15]. Age was assessed from the following question: “How old are you?” and finally only 17-30 years old females were analyzed. Body height and body weight were asked to the nearest 1 cm and 1 kg, respectively. BMI was calculated by body weight divided by the square of body height (kg/m^2^) [16]. Physical activity was accessed using “How often do you exercise in the past year?” Exercise was defined as continuous physical activity more than 30 mins per time. Having physical activity included those who choose “1-2 times a week or 3-4 times a week or 5-6 times a week or every day” while no physical activity includes those who chose “less than once a week.” Monthly expenditure was acquired by the following question “In the past year, how much do you cost monthly in average?” We divided participants into two parts, one was those who choose “≤2000RMB” and the other was those who choose “2001-4000RMB or 40001-8000RMB or 8001-15000 or >15000.” Medicine history was investigated by providing question: “Did you take medicine leading to menstruation irregularity in the past year, such as hormone or large dose of antibiotics” (yes or no).

### 2.3. Assessment

The main contents of the questionnaire are separated into two parts: sleep conditions and menstrual conditions. In investigations of sleep conditions, the respondents are primarily divided into two groups by the question:

Do you have the situations below?

- None
- Stay up late or occasionally insomnia
- Always insomnia (cannot fall asleep in 30 minutes more than three times a week for a month)
- Always stay up overnight (more than three times a week for one month)

If the respondent chose the first two options, they would be asked their specific sleep conditions: one's bedtime (before 00:00 or after 00:00), one's bedtime regularity (never break the bedtime, break it sometimes, or always break it), one's average sleep duration (in hours), and sleep quality (without any symptom, or have any one of the symptoms including difficulty initiating sleep, difficulty maintaining sleep, early morning awakening, dreaminess, and somnolent state). If the respondent chose the last two options, they would only be investigated their average sleep durations (average sum hours in one week and then calculated into daily duration), and sleep quality (same as above).

Secondly, the menstrual conditions of respondents are defined by questions: menstrual menarche (age), menstrual duration (day), menstrual volume (described below), menstrual cycle (≤25 days, 26-35 days, >35 days), self-awareness menstrual regularity (regular or irregular), and dysmenorrhea (yes or never). In particular, the numeric value of menstrual volume is calculated by the formula:

(1) $$\begin{array}{c} \text{Menstrual volume}=\text{Days of Light bleeding}\times 2.5\text{ ml}/\text{pad}\times 5\text{ pads}/\text{day}+\text{Days of Normal bleeding}\times 5\text{ ml}/\text{pad}\times 5\text{ pads}/\text{day}+\text{Days of Heavy bleeding}\times 10\text{ ml}/\text{pad}\times 5\text{ pads}/\text{day}. \end{array}$$

Therefore, the questionnaire inquired “the numbers of days” of light/normal/heavy bleeding with corresponding volume on pads (5 pads use per day) and showed the pictures of pads with 2.5 ml/5 ml/10 ml liquid (Figure 1).

### 2.4. Statistical Analyses

Descriptive statistics were obtained to describe the study population as a whole and divided in subgroups. Mean values and standard deviations (SD) were calculated for quantitative variables; frequency distributions were calculated for qualitative variables. Meanwhile, based on previous studies and mean ± SD, two categories were divided for menstrual cycle (normal: 26-35 days; abnormal: ≤25 days or >35 days).

Linear regression analyses and binary logistic regression analyses were used to examine the associations between bedtime, bedtime regularity, average sleep duration, sleep quality and menstrual cycle, self-awareness menstrual regularity, dysmenorrhea adjusting for the effects of physical status (age, BMI, physical activities, and medicine history), and socioeconomic covariates (monthly expenditure). The definitions of statistical analysis variables were shown in Supplementary Table 1. All statistical analyses were performed using IBM SPSS Statistics for Windows, Version 22.0 (Armonk, New York: IBM Corp.).

## 3. Results

### 3.1. Sample Characteristics

Of the 2517 individuals engaged in this survey, we excluded those aged ≤16 (*N* = 4) or >30 (*N* = 86), those height ≤ 1.40 m or ≥1.90 m (*N* = 4), those weight ≤ 30 kg or ≥90 kg (*N* = 15), those who slept for <4 hours (*N* = 3), those who smoked >1 cigarette per day (*N* = 7), those who were diagnosed tumor, cardiovascular disease, immune disease, urologic disease, diabetes, thyroid dysfunction, and gynecological disease (*N* = 32), those whose menarche age ≥ 19 (*N* = 7), and those with inconsistent and inaccurate data (*N* = 60). Finally, the data of 2260 young female were analyzed.

Mean age was 21.1 years old (SD = 2.46). 68.9% of participants consumed less than or equal to 2000 RMB per month, and 31.1% of participants consumed more than 2000 RMB monthly. In all sample, 31.5% of their BMI were lower than 18.5, 63.1% were in normal range of 18.5~24.9, and 5.3% were overweight. For whether they had habit of physical activities in the past year, 38.4% answered “No,” while 61.6% answered “Yes.” 86.9% of participants denied taking any medication that influenced menstruation in the past year; the rest gave a positive answer.  Table 1 summarizes basic information.

### 3.2. Menstrual Status and Sleep Status

Regarding self-awareness menstrual regularity, 28.9% of the female reported having irregular periods. More than 81.6% of the female reported having period pain. For menstrual cycle, 15.6% and 11.4% of female reported having abnormal menstrual cycle no more than 25 days and longer than 35 days, respectively. According to the result, mean menstrual volume of sample was 151.97 (SD = 42.70) ml. Mean sleep duration of the samples was 7.24 hours (SD = 0.92). In terms of sleep quality, 38.3% reported good sleep quality, and 61.7% were poor. For bedtime, 47.1% of participants sleep before 00:00, the rest after 00:00. Regarding bedtime regularity, 10.8% of samples reported never breaking the regularity, 78.4% breaking it sometimes, 1.7% always breaking the regularity, and 9.2% did not answer this question.  Table 1 summarizes menstrual status and sleep status.

### 3.3. Menstrual Blood Volume and Sleep Status

For effects of bedtime, bedtime regularity, sleep duration, and sleep quality on menstrual volume, see Table 2. For the entire sample, there was a significant association between menstrual volume and the regularity of bedtime, and this association was reflected in irregular bedtimes, with less menstrual volume (*B* = −6.140, *P* = 0.019). There was no significant association between menstrual flow and bedtime (*P* = 0.341), sleep time (*P* = 0.083), and sleep quality (*P* = 0.258).

### 3.4. Dysmenorrhea and Sleep Status

For effects of bedtime, bedtime regularity, sleep duration, and sleep quality ondysmenorrhea, see Table 3. For the entire sample, dysmenorrhea had no significant association with bedtime regularity (*P* = 0.060) and sleep duration (*P* = 0.738). Through binary logistic regression analysis (stepwise screening of independent variables), correcting age, BMI, monthly expenditure, physical exercise, and medication history, dysmenorrhea was positively correlated with bedtime (OR [95%CI] = 1.38 [1.16-1.64], *P* < 0.001) and sleep quality (OR [95%CI] = 1.74 [1.40-2.17], *P* < 0.001).

### 3.5. Menstrual Cycle and Sleep Status

For effects of bedtime, bedtime regularity, sleep duration, and sleep quality on menstrual cycle, see Table 4. For the entire sample, menstrual cycle had no significant association with bedtime (*P* = 0.975), bedtime regularity (*P* = 0.465), sleep duration (*P* = 0.192), and sleep quality (*P* = 0.415).

### 3.6. Self-Awareness Menstrual Regularity and Sleep Status

As presented in Table 5, relationship between self-awareness menstrual regularity and sleep status including bedtime, bedtime regularity, sleep duration, and sleep quality are shown. Self-awareness menstrual regularity was not associated with bedtime (*P* = 0.982), bedtime regularity (*P* = 0.582), and sleep duration (*P* = 0.808). However, by binary logistic regression analysis (stepwise screening of independent variables) and after correcting age, BMI, monthly expenditure, physical exercise, and medication history, self-awareness menstrual regularity was significantly correlated with sleep quality (OR [95%CI] = 1.29 [1.06-1.56], *P* = 0.006).

## 4. Discussion

This is a comprehensive study to examine sleep patterns, insomnia symptoms, and sleep quality in relation to menstrual symptoms and cycles in Chinese healthy, young, ovulating women. The statistical analysis revealed that sleep quality was a significantly associated factor with menstrual pain and menstrual regularity. These associations did not change even after adjusting for potential confounding factors including age, physical activity, BMI, monthly expenditure, and medications.

To the best of our knowledge, our study firstly investigated the importance of sleep patterns in relation to menstrual volume among Chinese females. The linear regression analysis showed that the bedtime regularity (*B* = −6.140, *P* = 0.019) was significantly associated with menstrual volume. In young women, the more frequent violations of schedules may be associated with less menstrual volume. The bedtime (*P* = 0.341), sleep duration (*P* = 0.083), or sleep quality (*P* = 0.258) were not significantly associated with menstrual volume, respectively. It needs more evidence to confirm relationships. The binary logistic analysis revealed that bedtime (OR [95%CI] = 1.38 [1.16-1.64], *P* < 0.001) and dysmenorrhea (OR [95%CI] = 1.74 [1.40-2.17], *P* < 0.001) were significantly associated with sleep quality. Factors such as bedtime regularity (*P* = 0.060) and sleep duration (*P* = 0.738) did not have associations with dysmenorrhea. In our questionnaire, the poor sleep quality was defined by suffering any of the following sleep problems: difficulty initiating sleep or insomnia (time of initiating sleep lasts more than 30 minutes), difficulty maintaining sleep, difficulty awakening or early morning awakening, dreaminess, and somnolence. As in our study, some prior studies [17, 18] reported that there were no significant associations between dysmenorrhea and factors such as sleep-work patterns, bedtime, and sleep durations, while the association between period pain and sleep quality was significant [19]. Similarly, a Korean study reported that there was a significant association between sleep disturbance and menstrual problems (*P* = 0.003) in Korean girls aged 12~18 years old [14].

There may be direct and indirect interactions between sleep disturbance and dysmenorrhea. For example, period pain and irregular periods are the leading causes of school absenteeism, which results in an increased risk of mental health problems and suicidality [7, 20, 21]. In turn, mental health problems worsen sleep quality. Yet, physiological mechanisms related these associations need further studies to give insights into the management of menstrual symptoms and sleep quality.

Our results showed that bedtime (*P* = 0.975), bedtime regularity (*P* = 0.465), sleep duration (*P* = 0.192), and sleep quality (*P* = 0.415) were not statistically associated with menstrual cycle interval. Bedtime (*P* = 0.982), bedtime regularity (*P* = 0.582), or sleep duration (*P* = 0.808) was not statistically associated with self-awareness menstrual regularity, either. However, our findings suggested that sleep quality was positively associated with menstrual regularity (OR [95%CI] = 1.29 [1.06-1.56], *P* = 0.011) through binary logistic regression analysis (stepwise screening independent variables), and the association did not change even after adjusting for potential confounding factors. The mechanism may be explained by effects of gonadotropins. Disrupted sleep inhibits luteinizing hormone secretion, and menstrual cycle irregularity may be linked with changes in luteinizing hormone pulsatility and amplitude, resulting from the disturbance of circadian rhythmicity and poor sleep quality. In a previous 12-month follow-up study, it showed that insomnia was associated with a 3.05-fold increase in the prevalence of menstrual cycle irregularity compared with not having insomnia after adjusting for age, BMI, and physical activity [22]. And that conclusion is consistent with our finding, which revealed that the sleep quality was positively correlated with menstrual regularity.

As mentioned before, the result did not show a significant association between sleep duration and menstrual regularity. However, a study showed that the sleep duration was associated with menstrual irregularities in Korean adolescents [23]. Another recent cross-sectional study highlighted that women who reported less than 6 h of sleep were more likely to have abnormal menstrual cycle lengths than women who slept more than 6 h [24]. These two conclusions were contrary to our result. The possible reason may be that their participants were from different countries, or our sample size was not large enough.

The present study has some limitations. First, this population-based study used retrospective self-report data, which could exist a potential for recall bias. Second, the causal relationship should be cautiously interpreted when identifying the relationships among variables due to the cross-sectional design of this study. Third, the data of subjects' menstrual cycle irregularity were self-reported, which may depend on subjective perceptions. Biomedical markers and hormone measurements need to be introduced to define menstrual cycle irregularity in future studies. Fourth, the calculated menstrual volume was larger than the published value. The possible reason might be that we used three pictures to show light, regular, and heavy blood loss, which is lack of a “spotting” level. Fifth, the assessment of menstrual symptoms lacks a standard scale, which imposes difficulties in comparisons. More studies were needed to establish a questionnaire scale to evaluate the menstrual health of females. Moreover, epidemiologic studies on the converse relationship between sleep disturbance and menstrual cycle irregularity are limited [17]. Biological and genetic mechanisms between women's sleeping status and menstrual problems need to be further studied.

## 5. Conclusions

In conclusion, women with poor sleep quality, whether mild or more severe levels, were more likely to have an irregular menstrual cycle and dysmenorrhea than those with good sleep quality. Putting together findings from previous studies and our study, public health providers should take into consideration the significance of the associations between sleep quality and menstrual regularity in females, and the significance of good sleep quality to prevent dysmenorrhea.

## Figures and Tables

**Figure 1:** Pads filled with different amount of bleeding fluid.

**Table 1:** Characteristics of included participants.

	*N* (%) or mean ± SD^∗^
*N*	2260 (100.0)
Age, years	21.13 ± 2.46
Monthly expenditure, RMB	
≤2000	1558 (68.9)
>2000	702 (31.1)
BMI, kg/m^2^	19.93 ± 2.76
BMI, kg/m^2^	
<18.5	713 (31.5)
>18.5, <25	1427 (63.1)
≥25	120 (5.3)
Physical activity, time/week	
<1	868 (38.4)
≥1	1392 (61.6)
Medication history, *N* (%)	
No	1964 (86.9)
Yes	296 (13.1)
Menarche age, years	12.83 ± 1.41
Menstrual duration, days	5.49 ± 1.28
Menstrual cycle interval, days	
≤25	353 (15.6)
26-35	1649 (73.0)
>35	258 (11.4)
Self-awareness menstrual regularity, *N* (%)	
Normal	1606 (71.1)
Abnormal	654 (28.9)
Menstrual volume, ml	151.97 ± 42.70
Dysmenorrhea, *N* (%)	
No	415 (18.4)
Yes	1845 (81.6)
Bedtime, *N* (%)	
Before 00:00	1065 (47.1)
After 00:00	988 (43.7)
Statistical missing	207 (9.2)
Bedtime regularity, *N* (%)	
Never break	243 (10.8)
Sometimes break	1771 (78.4)
Always break	39 (1.7)
Statistical missing	207 (9.2)
Sleep duration, h	7.24 ± 0.92
Sleep quality, *N* (%)	
Without symptoms^∗∗^	866 (38.3)
With symptoms^∗∗^	1394 (61.7)

^∗^SD = standard deviation; ^∗∗^symptoms include any of the following: difficulty initiating sleep, difficulty maintaining sleep, dreaminess, early morning awakening, and somnolence.

**Table 2:** Linear regression analysis of menstrual blood volume and sleep status.

	*B* ^∗^	SE^∗∗^	*t*	*P* value
Bedtime	1.327	1.392	0.953	0.341
Bedtime regularity	-6.140	2.613	-2.349	0.019
Sleep duration	1.757	1.015	1.732	0.083
Sleep quality	2.105	1.860	1.132	0.258

^∗^ *B* = regression coefficients; ^∗∗^SE = standard error.

**Table 3:** Logistic regression analysis of dysmenorrhea and sleep status.

	*B* ^∗^	SE^∗∗^	Wald^∗∗∗^	OR (95% CI)^∗∗∗∗^	*P* value
Bedtime	0.322	0.089	13.22	1.38 (1.16, 1.64)	<0.001
Bedtime regularity	0.288	0.153	3.53	1.33 (0.99, 1.80)	0.060
Sleep duration	0.021	0.062	0.112	1.02 (0.91, 1.15)	0.738
Sleep quality	0.556	0.111	25.23	1.74 (1.40, 2.17)	<0.001

^∗^ *B*: regression coefficients; ^∗∗^SE: standard error; ^∗∗∗^Wald: Chi-square value; ^∗∗∗∗^OR: odds ratio; CI: confidence interval.

**Table 4:** Logistic regression analysis of menstrual cycle and sleep status.

	*B* ^∗^	SE^∗∗^	Wald^∗∗∗^	OR (95% CI)^∗∗∗∗^	*P* value
Bedtime	0.002	0.074	0.001	1.00 (0.87, 1.16)	0.975
Bedtime regularity	-0.102	0.140	0.553	0.90 (0.69, 1.19)	0.465
Sleep duration	-0.072	0.055	1.702	0.93 (0.84, 1.04)	0.192
Sleep quality	0.081	0.099	0.665	1.08 (0.89, 1.32)	0.415

^∗^ *B*: regression coefficients; ^∗∗^SE: standard error; ^∗∗∗^Wald: Chi-square value; ^∗∗∗∗^OR: odds ratio; CI: confidence interval.

**Table 5:** Logistic regression analysis of sleep status and self-awareness menstrual regularity.

	*B* ^∗^	SE^∗∗^	Wald^∗∗∗^	OR (95% CI)^∗∗∗∗^	*P* value
Bedtime	0.002	0.072	<0.001	1.00 (0.87, 1.15)	0.982
Bedtime regularity	0.078	0.142	0.303	1.08 (0.82, 1.43)	0.582
Sleep duration	-0.013	0.054	0.059	0.99 (0.89, 1.10)	0.808
Sleep quality	0.251	0.099	6.452	1.29 (1.06, 1.56)	0.011

^∗^ *B*: regression coefficients; ^∗∗^SE: standard error; ^∗∗∗^Wald: Chi-square value; ^∗∗∗∗^OR: odds ratio; CI: confidence interval.

## Data Availability

Under reasonable circumstances, the survey data of this study can be obtained from the corresponding author via email.

## Abbreviations

BMI: Body mass index
SD: Standard deviations
SE: Standard error
OR: Odds ratio
CI: Confidence interval.

## Supplementary Materials

Supplementary Materials Supplementary Table 1: definitions of statistical analysis variables.
